# Clinical Characteristics and Treatment Overview in Hand-Foot-and-Mouth Disease Using Real-World Evidence Based on Hospital Information System

**DOI:** 10.1155/2022/9156186

**Published:** 2022-09-20

**Authors:** Guoming Chen, Chuyao Huang, Dongqiang Luo, Jiawei Yang, Yuzhen Shi, Danyun Li, Zhuoyao Li, Tie Song, Hua Xu, Fen Yang

**Affiliations:** ^1^Guangzhou University of Chinese Medicine, Guangzhou, China; ^2^School of Chinese Medicine, Li Ka Shing Faculty of Medicine, The University of Hong Kong, Hong Kong SAR, China; ^3^Guangdong Center for Disease Control and Prevention, Guangzhou, China; ^4^First Affiliated Hospital of Guangzhou University of Chinese Medicine, Guangzhou, China

## Abstract

**Objectives:**

To describe the epidemiological characteristics and medication overview of HFMD in Guangzhou and analyze the factors of length of stay (LOS) based on TCM usage.

**Method:**

From January 1, 2014, to June 30, 2019, clinical data of HFMD (ICD-10 B08.401) as the initial diagnosis, based on HIS of five medical institutions for outpatient and inpatient cases, was collected. The inpatient cases of the five hospitals in Guangzhou were utilized for hospitalization analysis. Information extracted from the warehouse was standardized. Descriptive analysis was used for baseline characteristics, medication usage, and inpatient characteristics. Potential factors were analyzed by bivariate analysis. COX regression analysis and Kaplan–Meier analysis for calculating HRs and 95% CIs were adopted to determine the predictors of LOS. Stratified COX regression was applied to analyze the relationship between predictors and LOS and to calculate interaction.

**Results:**

A total of 14172 patients with HFMD were included. It showed that HFMD would occur in males, infants, and summer. Cause and symptoms are the two aspects of conventional Western medicine treatments, while TCM treatment of HFMD took clearing heat and detoxification as the basic principle. Inpatients with HFMD were divided into two groups by the use ratio of TCM. Age, season, and disease severity were possible correlated factors of LOS, extrapolating from their disparity in distribution. By stratified Cox regression, three factors following presented as possible contributions to shortening LOS, including TCM ≥ 0.1 (HR = 1.79, 95% CI (1.67–1.92), *P* < 0.01), winter (HR = 1.28, 95% CI (1.12–1.47)), *P* < 0.01), mild HFMD (HR = 1.93, 95% CI (1.69–2.22), *P* < 0.01). Additive interaction of TCM use and disease severity was significant (RERI = 1.014 (0.493–1.534), *P* < 0.01).

**Conclusion:**

Young children and high temperature were the risk factors of HFMD infection, which suggests that increasing surveillance for susceptible particular-age individuals and season is indispensable. Favorable factors to decrease LOS included a higher proportion of TCM use, mild HFMD, and onset in winter. The proportion of TCM use had additive interaction with disease severity, indicating that TCM may have antiviral and other biological effects on HFMD. Increasing the proportion of TCM use was probably beneficial to shortening LOS.

## 1. Introduction

Hand-foot-and-mouth disease (HFMD) is a common contagion caused by picornaviruses, especially human enteroviruses and coxsackieviruses [1]. Due to its features of self-limiting, few concentrations have been put on this disease. And its identical clinical manifestations, presenting as a low-grade fever with a maculopapular or papulovesicular rash on the hands and soles of the feet and painful oral ulcerations, make it easy to be overlooked [2]. While in recent years, some evidence has shown that HFMD can also cause neurologic or cardiopulmonary complications, which can lead to poor prognosis or even death [3]. A 0.30% mortality was reported in China and it maintained a high recurrence rate from 2008 to 2014 [4]. Guangdong is a populous province in China, where rising morbidity of HFMD has been witnessed in recent years, making it a common infectious disease [5]. The timing of monitoring the susceptible population is of great significance for disease prevention.

Currently, a large sample of clinical data is still needed to support the optimal proposal of treatment. There has not been an approved antiviral treatment for HFMD, particularly for the causative virus [2]. While as suggested, mild HFMD should be managed according to the symptoms, whose primary therapeutic purpose is to relieve pain, abate fever, and stay hydrated [2]. And in severe cases, supportive treatment and symptomatic treatment are mainly applied to keep basic life signs. As for prevention, the vaccine seems to be the best measure to combat HFMD. In China, three kinds of vaccines have been identified to be safe and protective [6–8]. Within the system of terms of traditional Chinese medicine (TCM), HFMD is included in the category of plague, rashes related to contagion. TCM had been recommended by the China Ministry of Health in 2010 for the treatment of HFMD, for its safety and high curative effect [9]. TCM can be used alone for relieving HFMD, of which the plant extracts have been demonstrated to have anti-infection properties [10, 11]. Flavonoids can suppress viruses, including glycyrrhizin [12], chrysin [13], etc. However, the clinical efficacy of TCM is still limited and in most cases, we regard the improvement of clinical symptoms as a key indicator of discharge. Hence, the factor of the length of stay (LOS) is viewed as one of the primary categories to evaluate efficacy.

In this study, we collected cases whose first-listed diagnosis is HFMD from 5 hospitals in Guangzhou, Guangdong, China. Data were extracted from the Hospital Information System (HIS), which involves reservation registration, pharmacy management, hospitalization management system, and toll collection. Based on the statistical analysis results, we described the clinical characteristics and treatment of HFMD in Guangzhou and analyzed the factors of LOS based on TCM usage.

## 2. Methods

### 2.1. Data Set and Sample Selection

This cross-section study extracted clinical data of outpatient and inpatient cases with HFMD (ICD-10 B08.401) as the first diagnosis from HIS. The collecting time ranged from January 1, 2014, to June 30, 2019. Medical institutions included the First Affiliated Hospital of Guangzhou University of Chinese Medicine, Guangdong Second Provincial General Hospital, Guangdong Provincial Hospital of Traditional Chinese Medicine, Guangdong Provincial Maternal and Child Health Care Hospital, and Guangzhou Women and Children's Medical Center. Among these, Guangdong Provincial Hospital of Traditional Chinese Medicine and Guangdong Second Provincial General Hospital had only outpatients. The information collection of cases included personal details (gender, age, address, admission time, and medical ID), diagnosis, prescription, dosage, unit, usage, and frequency. Given that follow-up visits may affect total treatment, we retained the first-visit ID at the same hospital.

### 2.2. Data Standardization

As the exported case details varied in each hospital information system, the data was standardized for analysis. Year became a transformation unit for age. For diagnosis, HFMD identification and classification would refer to ICD-10 and guidelines for the diagnosis and treatment of HFMD (2018 version) [14]. The frequency of a single herb, drug, or Chinese patent medicine was denoted as one. According to the patient's prescription, the proportion of TCM use was recorded. Chinese patent medicine with the same composition but different dosage forms was defined as the same drug; Western medicine was standardized according to the chemical name; Traditional Chinese medicine pieces were referred to Chinese Pharmacopoeia (2020 version) for standardization. For seasonal onset analysis, the visit time was divided into spring (March, April, and May), summer (June, July, and August), autumn (September, October, and November), and winter (December, January, and February). To analyze the onset feature in different developmental stages, the age in the yearly unit was divided into neonate (0–1 month), infant (1 month-2 year), preschool (2–6 year), child (6–12 year), adolescent (12–18 year) and adult (>18 year) [15].

### 2.3. Statistical Analysis

All data analyses were performed by SPSS 23.0 and R software (version 4.0.5). Depending on whether the data followed a normal distribution, mean ± standard deviation (SD) or median (interquartile range (IQR)) were adopted to describe measurement data. Enumeration data were presented as frequency. Descriptive analysis was used for the overview description of baseline characteristics, drug use, and inpatient case characteristics. Potential factors were analyzed by bivariate analysis. Through the survminer and survival packages of R software, Cox regression analysis was used to calculate HRs and 95% CIs to determine the independent and significant predictors of inpatient of patients with HFMD. Kaplan–Meier analysis was used for evaluating the effect of predictors on the LOS of patients with HFMD. The interaction R package was used to calculate the additive and multiplicative interactions of the two factors, and the forest plot package was used to draw COX regression analysis. A *P* value <0.05 was considered statistically significant.

## 3. Results

### 3.1. Patient Demographics and Baseline Characteristics

A total of 14172 patients with HFMD as the first diagnosis were included. Male cases (62.14%) were more than female cases (37.86%). Infancy accounted for the largest proportion (53.71%), followed by preschool (41.14%). Summer was the season with a high incidence of HFMD. The majority of HFMD patients were treated as outpatients with no more than three visits (Table 1).

### 3.2. Medication Use of HFMD

The most frequent Chinese herb was Glycyrrhizae radix et rhizoma, a tonifying medical, when it is not processed, it has the additional effect of heat-clearing, detoxicating, and dispelling phlegm. From the perspective of Chinese herb efficacy, the treatment of HFMD mainly focused on lowering the fever, clearing heat, removing dampness, and reducing phlegm (Table 2). The main application of Chinese patent medicine was an external application and oral administration, where, aerosol inhalation is a method to disperse the tiny droplet drug to the nose or throat, which is frequently used in respiratory disease. It can be seen from the above that TCM has flexible dosage form selection in the treatment of HFMD (Table 3). As for the use of Western drug, antimicrobial drugs had the highest frequency, aiming to control viral infections and other infectious complications. Adrenocortical hormones exerted anti-inflammatory and antiallergic synergy. *M* receptor blockers and adrenoceptor agonists can smooth wheezing (Table 4).

### 3.3. Factors of Hospitalization Day in HFMD

3615 patients were enrolled in the COX regression and Kaplan–Meier analysis, including 2346 males and 1269 females, with an age ranging from 21 days to 25 years. The patients were divided into two groups according to the proportion of TCM use, and there were significant differences in the distribution of age, season, and disease between the two groups (Table 5). Univariate COX regression showed significant correlated factors with LOS, including the proportion of TCM use, disease distribution, specific age section (neonate, infant, preschool, and child), and specific season (summer and spring) (Table 6). Kaplan–Meier analysis showed that disease type and the proportion of TCM use correlated significantly with LOS (Figure 1). Due to the adults and adolescents involved with too less quantity, the data were excluded in stratified COX regression. Confounding factors were adjusted by using three models Model1 adjusted age and sex; Model2 adjusted age, sex, and season; Model3 adjusted age, sex, season, and disease. Stratified COX regression showed that three factors were statistically significant in shortening hospitalization stay, including TCM ≥ 0.1 (HR = 1.79, 95% CI (1.67–1.92), *P* < 0.01), winter (HR = 1.28, 95% CI (1.12–1.47)), *P* < 0.01), mild HFMD (HR = 1.93, 95% CI (1.69–2.22), *P* < 0.01) (Table 7). TCM ≥ 0.1, mild HFMD, and onset in winter were favorable factors in shortening LOS (Figure 2). It could be noted that HR of TCM ≥ 0.1 and winter decreased after the addition of disease severity in Model3, and the increased risk of LOS was 11% and 3%, respectively. Additive interaction of the proportion of TCM use and disease severity was significant (RERI = 1.014 (0.493–1.534), *P* < 0.01), while multiplicative interaction of them was not (RR = 1.13 (0.81–1.57), *P*=0.49).

## 4. Discussion

HFMD is prevalent in China and is affected by living environment and meteorological factors. In 2008, the outbreak of HFMD in China led to a public health crisis, and consequently, it was classified as a *C*-class notifiable communicable disease by the Ministry of Health of China. The incidence of Guangdong was 4 times the national average [16], and a Bayesian spatiotemporal model showed a higher relative risk in Pearl River Delta [17]. To induce an overview of the characteristics and treatment of HFMD, this study collected real-world evidence of HFMD in Guangzhou, Guangdong.

For the epidemiological factors, HFMD seemed to be correlated with gender, age, and season. The ratio of men to women approximately was 1.64 : 1, which is in accordance with the result of a previous study [16, 18]. The etiology of HFMD was enterovirus infection, primarily caused by enterovirus 71 (EV71) and coxsackievirus A16 (Cox A16) [19]. It was reported that the latent infectious rate of enterovirus in healthy males in China was higher than in females [20]. Boys under high temperatures were at a higher risk of HFMD on lag 0 days in the distributed lag nonlinear model, while girls had an increasingly cumulative risk of HFMD with increased lag days [21]. Infants and preschools also had a higher incidence risk of HFMD in this study. The age-specific onset varied geographically: 3–5 years old in northern China and 0–2 years old in southern China [22], which was generally consistent with the results of this study. As infancy has not fully developed, the poor self-protection ability may be one of the factors for the high susceptibility. Of note, preschool children gathered in kindergarten, which could increase the risk of mutual infection [22]. However, the lack of stratification of vaccination history in this study may influence the results. Temperature (10–25°C), humidity (70–90%), wind speed (< 2.5 m/s), and sunshine time (> 9 h) are the risk factors for HFMD [23]. In Guangzhou, the temperature of summer maintains to be above 25°C, while high humidity can increase droplet transmission, and long-time sunshine generally raises the day/night temperature. This may be the reason for the highest prevalence in summer. Except in winter, the temperature is kept above 10°C for a long time, providing favorable conditions for enterovirus survival.

For medication use, the treatment of HFMD included traditional Chinese medicine decoction, Chinese patent medication, and Western medicine. In TCM theory, HFMD belongs to the category of “plague warm and clip wet” and the TCM treatment of HFMD needs to follow the progression stages. At eruption, wind syndrome, and dyspnea collapse stages, the fundamental law of treatment is heat-clearing and detoxicating, flexibly coordinating resolving dampness, outthrusting the pathogen, and calming endogenous wind [14]. Our results showed that the use of Chinese herbs and oral Chinese patent medicine was corresponding with the TCM pathogenesis of HFMD. It has been verified that Forsythiae Fructus had a function of anti-inflammation, antivirus, antibacterial, and neuroprotection according to the literature so far [24]. The antiviral activities may originate from the phenolic acids of Forsythiae Fructus [25, 26]. The extraction of Pogostemonis Herba can inhibit influenza viral infection, contributing to the recovery of pneumonia [27, 28]. The efficacy of external application and aerosol inhalation of Chinese patent medication can basically relieve papulovesicular rash and oral ulcerations, but further clinical evidence is needed to support this. Antimicrobial drugs occupied the largest proportion of Western medicine. Due to the lack of specific medicine for the enterovirus, ribavirin was one of the common antiviral drugs in the treatment of HFMD in this study. Cephalosporin and penicillins were used to control bacterial infections. Adrenocortical hormone had an effect on anti-inflammation and controlling edema which was adopted in case of HFMD with high fever or encephalomyelitis, as appropriate. *M* receptor blockers and adrenoceptor agonis are effective in alleviating bronchospasm and dyspnea. It can be seen that clinical treatment was mainly divided into etiological treatment and symptomatic treatment. Fever for more than 3 days, lethargy, pathologic reflexes, and convulsions were risk factors for severe HFMD [29].

The proportion of TCM use, disease severity, and the particular season were the significant correlated factors with LOS based on univariate COX regression. Stratified COX regression showed that three factors were significantly beneficial to decrease LOS, including TCM ≥ 0.1 (HR = 1.79, 95% CI (1.67–1.92), *P* < 0.01), winter (HR = 1.28, 95% CI (1.12–1.47)), *P* < 0.01), mild HFMD (HR = 1.93, 95% CI (1.69–2.22), *P* < 0.01). This study collected the admission date of inpatients with HFMD. Given that HFMD was an acute febrile illness, the hospitalization date generally was close to the onset date. Consistent with the previous research, the relatively high temperature would be the potential risk of HFMD. Correspondingly, in the case of low temperatures in winter, the virus is not easy to survive, which was a favorable condition to promote recovery and shorten the LOS. A randomized controlled trial showed the defervescence time of rectal administration of TCM plus conventional therapy was significantly shorter than conventional therapy alone [10]. Compared to Western medicine, Reduning injection plus Western medicine could significantly lower the fever and shorten the time of rash disappearance in mild HFMD [30]. It was speculated that the increased proportion of TCM use could decrease LOS. In addition, stratified COX regression showed that the risk of increased LOS was 11% (TCM ≥ 0.1) and 3% (Winter) after disease severity was added to adjusted Model3. The mild HFMD could significantly shorten LOS. So additive interaction of the proportion of TCM use and disease severity was significant, while multiplicative interaction of them had no statistical significance. Addition is more reasonable than multiplication in analyzing biological interactions. There is biological synergy between the two factors with positive additive interaction [31]. This may suggest TCM affects the progression of HFMD through a biological mechanism. Glycyrrhizic acid (GA) is extracted from *Glycyrrhiza* uralensis Fisch and has an antivirus effect. GA dose-dependently blocked viral replication of EV71 and CVA16. However, the two antiviral mechanisms were distinct since GA inactivated CVA16 directly but its anti-EV71 effect was associated with events post virus cell entry [32].

In this study, the region, incidence factors, vaccination history, and clinical symptoms of HFMD were not subdivided, and the characteristics of HFMD depend on more demographic data supply. Due to the lack of symptoms comparison and biochemical indicators, it was not comprehensive to evaluate the efficacy of TCM on HFMD. Also, the hospital discharge was not totally equivalent to a cure, considering the possibility of being transferred to the hospital after discharge. And more indicator support is still in need to evidence the efficacy of TCM on HFMD.

## 5. Conclusion

Surveillance for young individuals and high-temperature periods may be beneficial to early prevention. TCM treatment is based on the law of clearing heat, detoxifying, and resolving dampness, with flexible dosage forms. However, its clinical efficacy needs support from more high-quality clinical studies. Western medication treatment was mainly antiviral treatment combined with symptomatic treatment. The increased proportion of TCM use, mild HFMD, and onset in winter were favorable factors in shortening LOS. The proportion of TCM use and disease severity had significant additive interaction, indicating that TCM use could affect the biological mechanism of HFMD and eventually influence the LOS.

## Figures and Tables

**Figure 1:** Kaplan–Meier for factors of hospitalization days of HFMD. (a) Comparison of gender. (b) Comparison of disease type. (c) Comparison of the proportion of TCM use).

**Figure 2:** The analysis between LOS and factors is based on a forest plot of stratified COX regression.

**Table 1:** Baseline characteristics.

Characteristic	Patients (*n*)
Gender	
Male	8807
Female	5365
Age, year	
Neonate	11
Infant	7612
Preschool	5830
Child	540
Adolescent	44
Adult	135
Visit time	
Spring (3–5)	3801
Summer (6–8)	4857
Autumn (9–11)	3680
Winter (12–2)	1834
Type of hospital	
Outpatient	10426
Inpatient	3746
Visit frequency	
1–3	14112
4–6	58
>6	2

**Table 2:** Chinese herb use (Top 10).

Rank	Herbal drug	Efficacy	Frequency (*n*)
1	Glycyrrhizae radix et rhizoma	Tonifying and replenishing	1871
2	Forsythiae Fructus	Heat-clearing, detoxicating	1545
3	Pogostemonis Herba	Resolving dampness	1155
4	Belamcandae Rhizoma	Heat-clearing, detoxicating	1060
5	Phragmitis Rhizoma	Heat-clearing and fire-purging	988
6	Lophatheri Herba	Heat-clearing and fire-purging	984
7	Coicis semen	Dampness-draining diuretic	829
8	Platycodonis Radix	Clearing and resolving heat-phlegm	711
9	Scutellariae Radix	Clearing heat and drying dampness	697
10	Menthae Haplocalycis Herba	Releasing the exterior with pungent-cool	693

**Table 3:** Chinese patent medicine use (Top 10).

Rank	Chinese patent medicine	Usage	Frequency (*n*)
1	Kangfu Xinye	External application	3619
2	Chushi zhiyang xiye	External application	1944
3	Kaihoujian penwuji	Aerosol inhalation	1473
4	Kouqiangyan penwuji	Aerosol inhalation	1379
5	Jian'er qingjie ye	Oral administration	1306
6	Fuganlin koufuye	Oral administration	1080
7	Sihuangxiaoyan xiji	External application	1023
8	Qingrejieduqushi keli	Oral administration	908
9	Fufang yuxingcao keli	Oral administration	751
10	Jinlian qingre Paotengpian	Oral administration	606

**Table 4:** Systemic medication use (TOP 10).

Rank	Treatment	Frequency (*n*)
1	Antiviral drug	3269
2	Cephalosporin	1929
3	Adrenocortical hormones	1732
4	Penicillins	1374
5	M Receptor blocker	1158
6	H2 receptor blocker	933
7	Adrenoceptor agonists	757
8	Benzodiazepines	721
9	Mucolytic agents	571
10	Antituberculous drugs	390

**Table 5:** Characteristics of HFMD patient group based on the proportion of TCM use.

		Proportion of TCM use		*P*
		TCM < 0.1 (*n* = 1698)	TCM ≥ 0.1 (*n* = 1917)	
Age	Neonate	2	2	<0.01
	Infant	1032	1227	
	Preschool	644	649	
	Child	17	40	
	Adolescent	1	1	
	Adult	2	0	

Sex	Male	1093	1253	0.53
	Female	605	664	

Season	Spring	483	495	<0.01
	Summer	669	725	
	Autumn	396	571	
	Winter	150	126	

Disease severity	Mild	1512	1872	<0.01
	Severe	186	45	

**Table 6:** Univariate COX regression results.

		Coef	HR	*P*	95% CI
Age	Adolescent				
	Neonate	2.50	12.15	0.01	(1.70, 86.89)
	Infant	1.50	4.47	0.04	(1.11, 18.07)
	Preschool	1.47	4.34	0.04	(1.07, 17.53)
	Child	1.57	4.82	0.03	(1.17, 19.94)
	Adult	0.53	1.70	0.60	(0.24, 12.12)

Sex	Male				
	Female	0.03	1.03	0.40	(0.96, 1.10)

Season	Autumn				
	Spring	−0.15	0.86	0.00	(0.79, 0.94)
	Summer	−0.14	0.87	0.00	(0.80, 0.95)
	Winter	0.12	0.12	0.09	(0.98, 1.28)

Proportion of TCM use	<0.1				
	≥0.1	0.64	0.53	0.00	(0.49, 0.56)

Disease condition	Mild				
	Severe	−0.83	0.44	0.00	(0.38, 0.50)

**Table 7:** The relationship of LOS and factors in a patient with HFMD.

Factors	Model1	Model2	Model3
TCM ≥ 0.1	1.90 (1.77–2.03)	1.90 (1.78–2.04)	1.79 (1.67–1.92)
Age			
Neonate and infant			
Preschool	0.99 (0.92–1.06)	0.98 (0.92–1.05)	0.96 (0.89–1.03)
Child	0.97 (0.74–1.26)	0.96 (0.74–1.26)	0.99 (0.76–1.28)
Sex (female)	1.03 (0.96–1.10)	1.03 (0.96–1.10)	1.03 (0.96–1.10)
Season			
Spring			
Summer		1.00 (0.92–1.09)	1.02 (0.94–1.11)
Autumn		1.10 (1.00–1.20)	1.09 (1.00–1.20)
Winter		1.31 (1.15–1.50)	1.28 (1.12–1.47)
Disease (Nonserious)			1.93 (1.69–2.22)
Additive interaction: RERI = 1.014 (0.493–1.534), *P* < 0.01;			
Multiplicative interaction: Disease^*∗*^TCM0.1 RR = 1.13 (0.81–1.57), *P*=0.49			

Model1: adjust age, sex; Model2: adjust age, sex, season; Model3: adjust age, sex, season, disease.

## Data Availability

The clinical data used to support the findings of this study were supplied by Fen Yang under license and so cannot be made freely available. Requests for access to these data should be made to Fen Yang, 160 Qunxian Road, Panyu District, Guangzhou, Guangdong (e-mails: 492242163@qq.com).
